The article "Inferences for Stress-Strength Reliability Model in the Presence of Partially Accelerated Life Test to Its Strength Variable" was published in 2022. Journal: Comput Intell Neurosci.

# Inferences for Stress-Strength Reliability Model in the Presence of Partially Accelerated Life Test to Its Strength Variable

**DOI:** 10.1155/2022/4710536

**Published:** 2022-03-18

**Authors:** Rashad M. El-Sagheer, Ahlam H. Tolba, Taghreed M. Jawa, Neveen Sayed-Ahmed

**Affiliations:** ^1^Mathematics Department, Faculty of Science, Al-Azhar University, Naser City 11884, Cairo, Egypt; ^2^Mathematics Department, Faculty of Science, Mansoura University, Mansoura 35516, Egypt; ^3^Department of Mathematics and Statistics, College of Science, P.O. Box 11099, Taif University, Taif 21944, Saudi Arabia

## Abstract

We focus on estimating the stress-strength reliability model when the strength variable is subjected to the step-stress partially accelerated life test. Based on the assumption that both stress and strength random variables follow Weibull distribution with a common first shape parameter, the inferences for this reliability system are constructed. The maximum likelihood, two parametric bootstraps, and Bayes estimates are obtained. Moreover, approximate confidence intervals, asymptotic variance-covariance matrix, and highest posterior density credible intervals are derived. A simulation study and application to real-life data are conducted to compare the proposed estimation methods developed here and also check the accuracy of the results.

## 1. Introduction

Stress-strength models have attracted many statisticians for many years due to their applicability in different and diverse areas such as engineering, economics, and quality control, and, in the last years, there have been numerous applications to medical and engineering problems.

In the last ten years, many authors have been interested in studying the application of the simple stress-strength reliability model, which is more handled theoretically and at the same time is more simple and applicable to implement in practice. This model of reliability contains a strength variable *X* and a stress variable *Y*, which is exposed to it. Such a system will properly function when *X* exceeds *Y*; namely, *R*=*P*(*X* > *Y*) denotes the reliability system. Many estimation studies of reliability system are considered by several statistician researchers under both complete and censored samples from different models, for example, exponential distribution under progressive type-II censoring by Saraçoğlu et al. [1], Weibull distribution under complete samples by Kundu and Gupta [2], Kumaraswamy distribution under upper record values by Nadar and Kızılaslan [3], Kumaraswamy distribution under progressive type-II censoring by Nadar et al. [4], Lomax distribution under record values by Mahmoud et al. [5], Burr X distribution under complete samples by Surles and Padgett [6], inverse Lindley distribution under complete samples by Sharma et al. [7], exponential and Weibull by Kumar and Siju [8], Weibull-Gamma distribution under progressively type-II censored samples by Mahmoud et al. [9], general exponential form distribution under complete samples by Mokhlis et al. [10], Rayleigh distribution under complete samples by Afshin [11], modified Weibull model under progressively type-II censored samples by Soliman et al. [12], Lindley distribution using progressively first-failure censoring by Kumar et al. [13], generalized inverted exponential distribution under progressively first-failure censoring by Krishna et al. [14], Kumaraswamy exponential distribution under progressively type-II censored samples by El-Sagheer and Mansour [15], Burr XII distribution under progressively first-failure censored samples by Saini et al. [16], and generalized Maxwell failure distribution under progressive first-failure censoring by Saini et al. [17].

The article "Inferences for Stress-Strength Reliability Model in the Presence of Partially Accelerated Life Test to Its Strength Variable" was published in 2022. Journal: Comput Intell Neurosci.

In previous reliability studies, it is evident that it is difficult to observe the lifetime of highly reliable components because few failures occur in a limited test time due to the very long lifetimes under normal test conditions. Therefore, to overcome this problem, we are looking for a catalyst for early failure of the components. Since testing under normal conditions takes a long time, then the development of accelerated life testing (ALT) or partially accelerated life test (PALT) is needed, where units are subjected to a more severe environment (increased or decreased stress levels) than the normal operating environment so that failures can be induced quickly. In this case, ALT or PALT allows experimenters to control higher stress levels to be used in the test.

In PALT, only part of the test components run under a higher stress level than the normal level, while all the test components run under a higher stress level in ALT. We use PALT when the acceleration factor is unknown, where items are examined at both normal and accelerated conditions. According to Nelson [18], there are three types of stress in PALT: constant stress, step stress, and progressive stress. In step-stress partially accelerated life test (S-SPALT), items are tested at a normal level; if it does not fail, then the stress will be changed at a certain time. This type allows the experimenter to select multiple stress factors, for instance, temperature, voltage stress, thermal and electrical cycling and shock, vibration, mechanical stress, and radiation in life testing.

Many authors have studied the inference based on the S-SPALT models for different probability distributions under various cases for censored or complete data, including Weibull by Zhang et al. [19] and Ismail [20], extended Weibull by Zhang and Shi [21], Burr type XII by Abd-Elfattah et al. [22], exponentiated exponential distribution by Abdel-Hamid and Al-Hussaini [23], Lomax by El-Sagheer and Ahsanullah [24], Gompertz by Ismail [25], modified Weibull by Mahmoud et al. [26], Kumaraswamy Inverse Weibull by El-Sagheer and Mohamed [27], and Weibull-Gamma by El-Sagheer et al. [28].

The article "Inferences for Stress-Strength Reliability Model in the Presence of Partially Accelerated Life Test to Its Strength Variable" was published in 2022. Journal: Comput Intell Neurosci.

Recently, in parallel with progress in engineering, technology, and manufacturing, the experimenters may want to investigate the stress-strength reliability in case the strength component of the reliability system is exposed to an ALT. In this paper, we study a simple stress-strength model *R*=*P*(*X* > *Y*) when the component strength exposes to S-SPALT. This system can be described as follows: such a system starts with the normal use condition of the strength variable *X* and stress variable *Y*. If the system does not fail before the prespecified time *τ*, then the strength variable *X* runs at an acceleration factor (*λ*). This model will help us to evaluate *R* when induced early failures to *X*. Moreover, force to failure on strength may help us to see the effect of change on *R* due to not only stress variable *Y* but also exposed stress by accelerating on strength variable *X*. For this reason, we consider the S-SPALT model introduced by DeGroot and Goel [29] for strength variable *X*.

The outline of the paper is as follows. In Section 2, assumptions of S-SPALT for the stress-strength reliability model are provided.  Section 3 deals with the maximum likelihood estimate and asymptotic confidence intervals. Two parametric bootstrap methods are proposed in Section 4. In a Bayes paradigm, estimation techniques have been assayed in Section 5. In Section 6, a simulation study is conducted to compare the proposed procedures. In Section 7, a real-life data example is presented to illustrate the application of the proposed inference procedures. Finally, a conclusion is furnished in Section 8.

## 2. Assumptions of S-SPALT for Reliability System

Suppose that *X* denote the lifetime of a test item as strength under S-SPALT can be determined, according to DeGroot and Goel [29], by the relation

(1) $$\begin{array}{c} X=\left\{\begin{array}{cc} T, & T\leq \tau ,\\ \tau +\frac{\left(T-\tau \right)}{\lambda }, & T>\tau , \end{array}\right) \end{array}$$

with probability density function (PDF)

(2) $$\begin{array}{c} f\left(x\right)=\left\{\begin{array}{cc} f_{1}\left(x\right), & x\leq \tau ,\\ f_{2}\left(x\right), & x>\tau , \end{array}\right) \end{array}$$

where *T* is the lifetime under normal use condition, *τ* is the time when stress is changed, and *λ* is the acceleration factor as *λ* > 1. Suppose *X* and *Y* are independent random variables following Weibull distribution (WD) with parameters (*α*, *β*_1_) and (*α*, *β*_2_), respectively, that is, *X* ~ *W*  *D*(*α*, *β*_1_) and *Y* ~ *W*  *D*(*α*, *β*_2_), where the parameter *α* is common and known, considering strength *X* under S-SPALT with the PDF *f*(*x*) and CDF *F*(*x*) and primary stress *Y* with PDF *g*(*y*) and CDF *G*(*y*). According to Çetinkaya [30], a partially accelerated life test implemented stress-strength reliability estimation can be written as

(3) $$\begin{array}{c} R=P\left(X>Y\right)\\ =\int_{0}^{\tau }\int_{0}^{x}f_{1}\left(x\right)g\left(y\right)\text{d}y\text{ d}x+\int_{\tau }^{\infty }\int_{0}^{x}f_{2}\left(x\right)g\left(y\right)\text{d}y\text{ d}x\text{.} \end{array}$$

The PDF of S-SPALT implemented strength variable *X* as suggested by DeGroot and Goel [29], which is given as follows:

(4) $$\begin{array}{c} f\left(x\right)=\left\{\begin{array}{cc} \alpha \beta_{1}x^{\alpha -1}e^{-\beta_{1}x^{\alpha }}, & x\leq \tau ,\\ \alpha \lambda \beta_{1}{\left[\tau +\lambda \left(x-\tau \right)\right]}^{\alpha -1}e^{-\beta_{1}{\left(\tau +\lambda \left(x-\tau \right)\right)}^{\alpha }}, & x>\tau , \end{array}\right) \end{array}$$

and CDF is given as follows:

(5) $$\begin{array}{c} F\left(x\right)=\left\{\begin{array}{cc} 1-e^{-\beta_{1}x^{\alpha }}, & x\leq \tau ,\\ 1-e^{-\beta_{1}{\left(\tau +\lambda \left(x-\tau \right)\right)}^{\alpha }}, & x>\tau . \end{array}\right) \end{array}$$

Also, the PDF and CDF of primary stress *Y* are given by

(6) $$\begin{array}{c} g\left(y\right)=\alpha \beta_{2}y^{\alpha -1}e^{-\beta_{2}y^{\alpha }},\\ G\left(y\right)=1-e^{-\beta_{2}y^{\alpha }},y>0. \end{array}$$

Then, by using equations (4) and (6) in equation (3), the reliability of such a system can be obtained as

(7) $$\begin{array}{c} R=P\left(X>Y\right)\\ =\frac{\beta_{2}}{\beta_{1}+\beta_{2}}\left[1+\frac{1-\lambda }{\lambda +\beta_{2}/\beta_{1}}e^{-\tau^{\alpha }\left(\beta_{1}+\beta_{2}\right)}\right]. \end{array}$$

Then, if we put *α*=1 and *β*_*i*_=1/*θ*_*i*_, *i*=1,2, the reliability of such a system, *R*=*P*(*X* > *Y*), devolves to one-parameter exponential distribution. If *λ*=1, equation (7) becomes the reliability for a simple stress-strength system without any acceleration. From Figures 1 and 2, we notice the following: (i) The reliability of the system increases with increasing stress change time *τ*, when the acceleration factor *λ* is fixed. (ii) Increasing on acceleration factor *λ* reduces the reliability quickly.

The article "Inferences for Stress-Strength Reliability Model in the Presence of Partially Accelerated Life Test to Its Strength Variable" was published in 2022. Journal: Comput Intell Neurosci.

In equation (7), *α* is common and known, *τ* is the predetermined stress change time, and *β*_1_, *β*_2_, and *λ* are unknown and need to be estimated; then

(8) $$\begin{array}{c} R=P\left(X>Y\right)\\ =Q\left(\beta_{1},\beta_{2},\lambda \right). \end{array}$$

## 3. Maximum Likelihood Inference

Let *X*_1_, *X*_2_,…, *X*_*n*_ be a random sample of strength from *W*  *D*(*α*, *β*_1_) and *Y*_1_, *Y*_2_,…, *Y*_*m*_ be a random sample of stress from *W*  *D*(*α*, *β*_2_). Then, by considering equations (4) and (6), the likelihood function of observed samples in this reliability system is given by (see Çetinkaya [30])

(9) $$\begin{array}{c} L\left(\alpha ,\beta_{1},\beta_{2},\lambda |x,y\right)\\ =\prod_{i=1}^{r}\alpha \beta_{1}x_{\left(i\right)}^{\left(\alpha -1\right)}\exp\left\{-\beta_{1}x_{\left(i\right)}^{\alpha }\right\}\prod_{i=1}^{m}\alpha \beta_{2}y_{\left(i\right)}^{\alpha -1}\exp\left\{-\beta_{2}y_{\left(i\right)}^{\alpha }\right\}\prod_{i=r+1}^{n}\alpha \lambda \beta_{1}{\left[\tau +\lambda \left(x_{\left(i\right)}-\tau \right)\right]}^{\alpha -1}\exp\left\{-\beta_{1}{\left[\tau +\lambda \left(x_{\left(i\right)}-\tau \right)\right]}^{\alpha }\right\}, \end{array}$$

and equally

(10) $$\begin{array}{c} L\left(\alpha ,\beta_{1},\beta_{2},\lambda \right)\\ =\alpha^{\left(n+m\right)}\beta_{1}^{n}\beta_{2}^{m}\lambda^{\left(n-r\right)}\exp\left\{\left(\alpha -1\right)\left(\sum_{i=1}^{r}\log\;x_{\left(i\right)}+\sum_{i=r+1}^{n}\log\left[\tau +\lambda \left(x_{\left(i\right)}-\tau \right)\right]+\sum_{i=1}^{m}\log\;y_{\left(i\right)}\right)\right\}\exp\left\{-\beta_{1}\left(\sum_{i=1}^{r}x_{\left(i\right)}^{\alpha }+\sum_{i=r+1}^{n}{\left[\tau +\lambda \left(x_{\left(i\right)}-\tau \right)\right]}^{\alpha }\right)-\beta_{2}\sum_{i=1}^{m}y_{\left(i\right)}^{\alpha }\right\}. \end{array}$$

Hence, the logarithm of the likelihood function may then be written as

(11) $$\begin{array}{c} \ell \left(\alpha ,\beta_{1},\beta_{2},\lambda \right)=\left(n+m\right)\log\;\alpha +n\;\log\;\beta_{1}+m\;\log\;\beta_{2}+\left(n-r\right)\log\;\lambda \\ +\left(\alpha -1\right)\left(\sum_{i=1}^{r}\log\;x_{\left(i\right)}+\sum_{i=r+1}^{n}\log\left[\tau +\lambda \left(x_{\left(i\right)}-\tau \right)\right]+\sum_{i=1}^{m}\log\;y_{\left(i\right)}\right)\\ -\beta_{1}\left(\sum_{i=1}^{r}x_{\left(i\right)}^{\alpha }+\sum_{i=r+1}^{n}{\left[\tau +\lambda \left(x_{\left(i\right)}-\tau \right)\right]}^{\alpha }\right)-\beta_{2}\sum_{i=1}^{m}y_{\left(i\right)}^{\alpha }. \end{array}$$

Taking the first partial derivatives of the log-likelihood in (11) with respect to *β*_1_, *β*_2_, and *λ*, we get

(12) $$\begin{array}{c} \frac{\partial \ell }{\partial \beta_{1}}=\frac{n}{\beta_{1}}-\sum_{i=1}^{r}x_{\left(i\right)}^{\alpha }-\sum_{i=r+1}^{n}{\left[\tau +\lambda \left(x_{\left(i\right)}-\tau \right)\right]}^{\alpha }, \end{array}$$

(13) $$\begin{array}{c} \frac{\partial \ell }{\partial \lambda }=\frac{n-r}{\lambda }+\left(\alpha -1\right)\sum_{i=r+1}^{n}\frac{x_{\left(i\right)}-\tau }{\tau +\lambda \left(x_{\left(i\right)}-\tau \right)}-\alpha \beta_{1}\sum_{i=r+1}^{n}{\left[\tau +\lambda \left(x_{\left(i\right)}-\tau \right)\right]}^{\left(\alpha -1\right)}\left(x_{\left(i\right)}-\tau \right), \end{array}$$

where *r* ≠ 0 and *r* ≠ *n*. To get the MLEs of the unknown parameters, denoted by ${\hat{\beta }}_{1}$, ${\hat{\beta }}_{2}$, and $\hat{\lambda }$, we should equate ∂*ℓ*/∂*β*_1_, ∂*ℓ*/∂*β*_2_, and ∂*ℓ*/∂*λ* to zero; thus,

(14) $$\begin{array}{c} {\hat{\beta }}_{1}=n{\left[\sum_{i=1}^{r}x_{\left(i\right)}^{\alpha }+\sum_{i=r+1}^{n}{\left[\tau +\lambda \left(x_{\left(i\right)}-\tau \right)\right]}^{\alpha }\right]}^{-1}, \end{array}$$

(15) $$\begin{array}{c} \frac{n-r}{\hat{\lambda }}+\left(\alpha -1\right)\sum_{i=r+1}^{n}\frac{x_{\left(i\right)}-\tau }{\tau +\hat{\lambda }\left(x_{\left(i\right)}-\tau \right)}-\alpha {\hat{\beta }}_{1}\sum_{i=r+1}^{n}{\left[\tau +\hat{\lambda }\left(x_{\left(i\right)}-\tau \right)\right]}^{\left(\alpha -1\right)}\left(x_{\left(i\right)}-\tau \right)=0. \end{array}$$

Then, we use the Newton–Raphson iteration method to solve (15). Therefore, the MLE of *R*, denoted by ${\hat{R}}_{ML}$, can be obtained by considering the invariance property of the MLEs by replacing the parameters with their estimates as follows:

(16) $$\begin{array}{c} {\hat{R}}_{ML}=\frac{{\hat{\beta }}_{2}}{{\hat{\beta }}_{1}+{\hat{\beta }}_{2}}\left[1+\frac{1-\hat{\lambda }}{\hat{\lambda }+{\hat{\beta }}_{2}/{\hat{\beta }}_{1}}e^{-\tau^{\alpha }\left({\hat{\beta }}_{1}+{\hat{\beta }}_{2}\right)}\right], \end{array}$$

where the parameter *α* is common and known.

The article "Inferences for Stress-Strength Reliability Model in the Presence of Partially Accelerated Life Test to Its Strength Variable" was published in 2022. Journal: Comput Intell Neurosci.

### 3.1. Asymptotic Confidence Interval

In this subsection, we construct an asymptotic confidence interval (ACI) for *R* based on the asymptotic normal property of MLEs. Let $\hat{\delta }=\left({\hat{\beta }}_{1},{\hat{\beta }}_{2},\hat{\lambda }\right)$ be the MLEs of *δ*=(*β*_1_, *β*_2_, *λ*); according to Cohen [31], the observed Fisher information matrix, denoted by $I\left(\hat{\delta }\right)$, is defined by

(17) $$\begin{array}{c} I\left(\delta \right)=\left[I_{ij}\right]\\ ={\left[-\frac{\partial^{2}\ell }{\partial \delta_{i}\partial \delta_{j}}\right]}_{\delta =\hat{\delta }},\;i,j=1,2,3, \end{array}$$

where

(18) $$\begin{array}{c} I_{11}=\frac{-n}{\beta_{1}^{2}},\\ I_{12}=I_{21}=I_{23}=I_{32}=0,\\ I_{13}=I_{31}=-\alpha \sum_{i=r+1}^{n}{\left[\tau +\lambda \left(x_{\left(i\right)}-\tau \right)\right]}^{\left(\alpha -1\right)}\left(x_{\left(i\right)}-\tau \right), \end{array}$$

(19) $$\begin{array}{c} I_{33}=\frac{-\left(n-r\right)}{\lambda }-\left(\alpha -1\right)\sum_{i=r+1}^{n}\frac{{\left(x_{\left(i\right)}-\tau \right)}^{2}}{{\left[\tau +\lambda \left(x_{\left(i\right)}-\tau \right)\right]}^{2}}-\alpha \left(\alpha -1\right)\beta_{1}\sum_{i=r+1}^{n}{\left[\tau +\lambda \left(x_{\left(i\right)}-\tau \right)\right]}^{\left(\alpha -2\right)}{\left(x_{\left(i\right)}-\tau \right)}^{2}. \end{array}$$

Also, the variance of *R* is obtained by using the delta method as follows:

(20) $$\begin{array}{c} \sigma_{R}^{2}={\left(\frac{\partial R}{\partial \beta_{1}}\right)}^{2}I_{11}^{-1}+{\left(\frac{\partial R}{\partial \beta_{2}}\right)}^{2}I_{22}^{-1}+{\left(\frac{\partial R}{\partial \lambda }\right)}^{2}I_{33}^{-1}+2\left(\frac{\partial R}{\partial \beta_{1}}\right)\left(\frac{\partial R}{\partial \lambda }\right)I_{13}^{-1}, \end{array}$$

where the first partial derivatives included in (20) can be easily obtained and *I*_*ij*_^−1^ is the *ij* − th element of the inverse of the information matrix *I*(*δ*) as given by

(21) $$\begin{array}{c} I^{-1}\left(\delta \right)=\frac{1}{\left|I\left(\delta \right)\right|}\left(\begin{array}{ccc} \Lambda_{11} & 0 & \Lambda_{13}\\ \; & \Lambda_{22} & 0\\ \; & \; & \Lambda_{33} \end{array}\right), \end{array}$$

where |*I*(*δ*)|=*I*_11_*I*_22_*I*_33_ − *I*_22_*I*_13_^2^, Λ_11_=*I*_22_*I*_33_, Λ_13_=−*I*_13_*I*_22_, Λ_22_=*I*_11_*I*_33_ − *I*_13_^2^, and Λ_33_=*I*_11_*I*_22_. Therefore, the 100(1 − *γ*)% ACI of *R* is constructed as

(22) $$\begin{array}{c} \left(R-z_{\gamma /2}\sigma_{R},R+z_{\gamma /2}\sigma_{R}\right), \end{array}$$

where *z*_*γ*_ is 100(1 − *γ*)th upper percentile of standard normal variate *N*(0,1).

## 4. Parametric Bootstrap

In this section, we propose a resampling technique, the bootstrap procedure, to obtain a more widely used confidence interval. DiCiccio and Efron [32] introduced the bootstrap method and showed that the bootstrap method can improve the accuracy of the confidence intervals, especially when the sample is small such that the normal approximation is inappropriate. Besseris [33] showed that the bootstrap method can provide tighter confidence intervals. Reiser et al. [34] compared difference bootstrap confidence intervals by applying Monte Carlo simulation. Here, we study two bootstrap methods: bootstrap-p and bootstrap-t. These bootstrap confidence intervals work as follows.

### 4.1. Bootstrap-p

(1) Generate random samples *x*_1_, *x*_2_,…, *x*_*n*_ from *F*(*x*) and *y*_1_, *y*_2_,…, *y*_*m*_ from *G*(*y*) in (5) and (6), respectively. Calculate the MLEs of ${\hat{\beta }}_{1}$, ${\hat{\beta }}_{2}$, and $\hat{\lambda }$.
(2) Use ${\hat{\beta }}_{1}$, ${\hat{\beta }}_{2}$, and $\hat{\lambda }$ to generate independent bootstrap samples *x*_1_^*∗*^, *x*_2_^*∗*^,…, *x*_*n*_^*∗*^ from *F*(*x*) and *y*_1_^*∗*^, *y*_2_^*∗*^,…, *y*_*m*_^*∗*^ from *G*(*y*). Calculate the MLEs of unknown parameters based on the bootstrap samples, denoted by ${\hat{\beta }}_{1}^{*}$, ${\hat{\beta }}_{2}^{*}$, and ${\hat{\lambda }}^{*}$.
(3) Calculate the bootstrap estimate of *R* in (16), and denote by ${\hat{R}}^{*}$.
(4) Repeat Steps 2 and 3 *N* times; then we have $\left({\hat{R}}_{\left(1\right)}^{*},{\hat{R}}_{\left(2\right)}^{*},\ldots ,{\hat{R}}_{\left(N\right)}^{*}\right)$.
(5) Let $\varphi \left(x\right)=P\left({\hat{R}}^{*}\leq x\right)$ be the CDF of ${\hat{R}}^{*}$. Define ${\hat{R}}_{\text{boot}-p}\left(x\right)=\varphi^{-1}\left(x\right)$ for given *x*. Then, two-side 100(1 − *γ*)% percentile confidence intervals of *R* are given by
  (23) $$\begin{array}{c} \left[{\hat{R}}_{\text{boot}-p}\left(\frac{\gamma }{2}\right),{\hat{R}}_{\text{boot}-p}\left(1-\frac{\gamma }{2}\right)\right]. \end{array}$$

The article "Inferences for Stress-Strength Reliability Model in the Presence of Partially Accelerated Life Test to Its Strength Variable" was published in 2022. Journal: Comput Intell Neurosci.

### 4.2. Bootstrap-t

(1) The same as the bootstrap-p.
(2) The same as the bootstrap-p.
(3) The same as the bootstrap-p.
(4) Obtain the *t*_*R*_^*∗*^-statistics $t_{R}^{*}=\left({\hat{R}}^{*}-\hat{R}\right)/\sigma_{R}^{*}$, where *σ*_*R*_^*∗*^ given in (20).
(5) Repeat Steps 2, 3, and 4 *M* times; then we have (*t*_*R*_^*∗*(1)^, *t*_*R*_^*∗*(2)^,…, *t*_*R*_^*∗*(*M*)^).
(6) Let *ψ*(*x*)=*P*(*t*_*R*_^*∗*^ ≤ *x*) be the CDF of *t*_*R*_^*∗*^. Define ${\hat{R}}_{\text{boot}-t}\left(x\right)=\hat{R}+\psi^{-1}\left(x\right)\sigma_{R}$ for given *x*. Then, two-side 100(1 − *γ*)% bootstrap-t confidence intervals of *R* are given by
  (24) $$\begin{array}{c} \left[{\hat{R}}_{\text{boot}-t}\left(\frac{\gamma }{2}\right),{\hat{R}}_{\text{boot}-t}\left(1-\frac{\gamma }{2}\right)\right]. \end{array}$$

## 5. Bayes Estimation

Bayes estimation is quite different from MLE and bootstrap methods because it takes into consideration both the information from observed sample data and the prior information. It can characterize the problems more rationally and reasonably. Assume that both parameters *β*_1_ and *β*_2_ have independent Gamma priors, while the parameter *λ* has usual noninformative prior; see Carlin and Louis [35]:

(25) $$\begin{array}{c} \pi_{1}\left(\beta_{1}\right)\propto \beta_{1}^{a_{1}-1}e^{-b_{1}\beta_{1}},\;a_{1},b_{1}>0, \end{array}$$

(26) $$\begin{array}{c} \pi_{3}\left(\lambda \right)=\frac{1}{\lambda },\;\lambda >1. \end{array}$$

Here, *a*_1_, *a*_2_, *b*_1_, and *b*_2_ are the hyperparameters that reflect the prior knowledge about the unknown parameters. The joint prior of the unknown parameters *β*_1_, *β*_2_, and *λ* is then given by

(27) $$\begin{array}{c} \pi \left(\beta_{1},\beta_{2},\lambda \right)\propto \beta_{1}^{a_{1}-1}\beta_{2}^{a_{2}-1}\lambda^{-1}e^{-b_{1}\beta_{1}-b_{2}\beta_{2}}. \end{array}$$

Via Bayes' theorem, based on the considered joint prior (27) and the likelihood (10), the posterior distribution of *β*_1_, *β*_2_, and *λ* given data takes the form

(28) $$\begin{array}{c} \pi^{*}\left(\beta_{1},\beta_{2},\lambda |x,y\right)\propto \beta_{1}^{n+a_{1}-1}\beta_{2}^{m+a_{2}-1}\lambda^{n-r-1}e^{-b_{1}\beta_{1}-b_{2}\beta_{2}}\\ \times \prod_{i=r+1}^{n}{\left[\tau +\lambda \left(x_{\left(i\right)}-\tau \right)\right]}^{\alpha -1}\exp\left\{-\beta_{1}{\left[\tau +\lambda \left(x_{\left(i\right)}-\tau \right)\right]}^{\alpha }\right\}\times \prod_{i=1}^{r}\exp\left\{-\beta_{1}x_{\left(i\right)}^{\alpha }\right\}\prod_{i=1}^{m}\exp\left\{-\beta_{2}y_{\left(i\right)}^{\alpha }\right\}. \end{array}$$

It is clear that the conditional posterior densities of *β*_1_, *β*_2_, and *λ* can be written as

(29) $$\begin{array}{c} \pi_{1}^{*}\left(\beta_{1}|\beta_{2},\lambda ;x,y\right)=\beta_{1}^{n+a_{1}-1}\exp\left\{-\beta_{1}\left(\sum_{i=1}^{r}x_{\left(i\right)}^{\alpha }+\sum_{i=r+1}^{n}{\left[\tau +\lambda \left(x_{\left(i\right)}-\tau \right)\right]}^{\alpha }+b_{1}\right)\right\}, \end{array}$$

(30) $$\begin{array}{c} \pi_{2}^{*}\left(\beta_{2}|\beta_{1},\lambda ;x,y\right)=\beta_{2}^{m+a_{2}-1}\exp\left\{-\beta_{2}\left(\sum_{i=1}^{m}y_{\left(i\right)}^{\alpha }+b_{2}\right)\right\}, \end{array}$$

(31) $$\begin{array}{c} \pi_{3}^{*}\left(\lambda |\beta_{1},\beta_{2};x,y\right)=\lambda^{n-r-1}\prod_{i=r+1}^{n}{\left[\tau +\lambda \left(x_{\left(i\right)}-\tau \right)\right]}^{\alpha -1}\exp\left\{-\beta_{1}{\left[\tau +\lambda \left(x_{\left(i\right)}-\tau \right)\right]}^{\alpha }\right\}. \end{array}$$

Thus, under the squared error loss function, the Bayes estimate of *R*, denoted by ${\hat{R}}_{MC}$, can be obtained as the mean of the posterior function as given in the following:

(32) $$\begin{array}{c} {\hat{R}}_{MC}=\int_{1}^{\infty }\int_{0}^{\infty }\int_{0}^{\infty }Q\left(\beta_{1},\beta_{2},\lambda \right)\pi^{*}\left(\beta_{1},\beta_{2},\lambda |x,y\right)d\beta_{1}d\beta_{2}d\lambda . \end{array}$$

From (29) and (30), the full conditional posterior densities of *β*_1_ and *β*_2_ are Gamma(*n*+*a*_1_, ∑_*i*=1_^*r*^*x*_(*i*)_^*α*^+∑_*i*=*r*+1_^*n*^[*τ*+*λ*(*x*_(*i*)_ − *τ*)]^*α*^+*b*_1_) and Gamma(*m*+*a*_2_, ∑_*i*=1_^*m*^*y*_(*i*)_^*α*^+*b*_2_), respectively. Thus, the samples of *β*_1_ and *β*_2_ can be generated by using any Gamma routine. On the other hand, the expression of *π*_3_^*∗*^(*λ|β*_1_, *β*_2_; **x**, **y**) cannot be written as any well-known distribution. One can use the method proposed by Devroye [36] to generate sample data from this distribution.

The article "Inferences for Stress-Strength Reliability Model in the Presence of Partially Accelerated Life Test to Its Strength Variable" was published in 2022. Journal: Comput Intell Neurosci.

However, the Metropolis–Hastings (MH) with the Gibbs sampling scheme by using normal proposal *N*(., .) can be effectively used to simulate random samples from (25)–(27). The MH algorithm and Gibbs sampler work as follows:

(1) Use the MLEs as the initial value, denoted by ${\hat{\beta }}_{1}^{\left(0\right)},{\hat{\beta }}_{2}^{\left(0\right)},{\hat{\lambda }}^{\left(0\right)}$
(2) Set *i*=1
(3) Generate *β*_1_^(*i*)^ from Gamma(*n*+*a*_1_, ∑_*i*=1_^*r*^*x*_(*i*)_^*α*^+∑_*i*=*r*+1_^*n*^[*τ*+*λ*(*x*_(*i*)_ − *τ*)]^*α*^+*b*_1_)
(4) Generate *β*_2_^(*i*)^ from Gamma(*m*+*a*_2_, ∑_*i*=1_^*m*^*y*_(*i*)_^*α*^+*b*_2_)
(5) Using MH algorithm,
  (i) Generate *λ*^*∗*^ from the proposal normal distribution *N*(*λ*^(*i* − 1)^, Var(*λ*)).
  (ii) Evaluate the acceptance probabilities
    (33) $$\begin{array}{c} \Omega_{\lambda }=\min\left[1,\frac{\pi_{3}^{*}\left(\lambda^{*}|\beta_{1}^{\left(i\right)},\beta_{2}^{\left(i\right)};x,y\right)}{\pi_{3}^{*}\left(\lambda^{\left(i-1\right)}|\beta_{1}^{\left(i\right)},\beta_{2}^{\left(i\right)};x,y\right)}\right]. \end{array}$$
  (iii) Generate *u* from Uniform (0,1) distribution.
  (iv) If *u* < Ω_*λ*_, accept the proposal and set *λ*^*∗*^=*λ*^(*i*)^; else set *λ*^(*i*)^=*λ*^(*i* − 1)^.
(6) Compute *R*_MC_^(*i*)^ at *β*_1_^(*i*)^, *β*_2_^(*i*)^, and *λ*^(*i*)^
(7) Set *i*=*i*+1
(8) Repeat Steps 3 − 10 *N* times and obtain *R*_MC_^(*i*)^, *i*=1,2,…, *N*

Then, the Bayesian estimators of ${\hat{R}}_{\text{MC}}$ under the squared error loss function are given by

(34) $$\begin{array}{c} {\hat{R}}_{\text{MC}}=\frac{1}{N-N_{0}}\sum_{i=M+1}^{N}R_{\text{MC}}^{\left(i\right)}, \end{array}$$

where *N*_0_ is burn-in to guarantee the convergence and to remove the affection of the selection of initial values. Therefore, the 100(1 − *γ*)% highest posterior density (HPD) Bayes credible interval is given by

(35) $$\begin{array}{c} {\hat{R}}_{\text{MC}\left[\gamma /2\left(N-N_{0}\right)\right]},{\hat{R}}_{\text{MC}\left[\left(1-\gamma /2\right)\left(N-N_{0}\right)\right]}. \end{array}$$

## 6. Simulation Study

In this section, we apply a Monte Carlo simulation to assess the performance of MLEs, bootstrap, and Bayes estimator methods for the stress-strength reliability model with component strength under PALT, along with their ACIs, bootstrap CIs, and HPD credible intervals. Furthermore, we study the variations on reliability with the different cases for both acceleration factor *λ* and stress change time *τ*. The performance of estimators is evaluated in terms of mean square error (MSE) for the point estimates, also coverage probability (CP), and average lengths (ALs) for interval estimates (asymptotic, bootstrap, and HPD). We consider five sample sizes such as (*n*, *m*)=(10,15), (20,25), (40,45), (60,60), and (90,90) for eight cases of the true values of the parameters, stress change times, acceleration factor, and corresponding actual values of *R*, when the common parameter *α*=2. These cases are as follows:

**Case 1 .**

*β*_1_=0.4, *β*_2_=2, *τ*=0.5, *λ*=2, and *R*=0.76799.

The article "Inferences for Stress-Strength Reliability Model in the Presence of Partially Accelerated Life Test to Its Strength Variable" was published in 2022. Journal: Comput Intell Neurosci.

**Case 2 .**

*β*_1_=0.4, *β*_2_=2, *τ*=1.25, *λ*=5, and *R*=0.82549.

**Case 3 .**

*β*_1_=0.4, *β*_2_=2, *τ*=1.5, *λ*=3, and *R*=0.8323.

**Case 4 .**

*β*_1_=0.4, *β*_2_=2, *τ*=2, *λ*=3, and *R*=0.8333.

**Case 5 .**

*β*_1_=2.5, *β*_2_=1.5, *τ*=0.4, *λ*=2, and *R*=0.2989.

**Case 6 .**

*β*_1_=2.5, *β*_2_=1.5, *τ*=1.5, *λ*=2, and *R*=0.3749.

**Case 7 .**

*β*_1_=2.5, *β*_2_=1.5, *τ*=0.4, *λ*=4, and *R*=0.3092.

**Case 8 .**

*β*_1_=2.5, *β*_2_=1.5, *τ*=1.5, *λ*=4, and *R*=0.3750.

The first four cases provide us with the upper (around 0.81477) actual values of *R* and their outcomes presented in Tables 1–4, while the second four cases provide us with the lower (around 0.3395) actual values of *R* and their results are given in Tables 5–8. The study is performed for 1000 replicates. For each replication, 1000 bootstrap samples are used. The Bayes estimates and the credible intervals are computed based on 12000 MCMC samples and discard the first values 2000 as “burn-in.” For Bayesian analysis, we consider informative prior with hyperparameters values *a*_1_=2, *b*_1_=1, *a*_2_=2, and *b*_2_=1. The results of this study are reported in Tables 1–8. In the first rows of these tables, the estimates and their ACIs are given, respectively, for all sample sizes (*n*, *m*). Besides, the MSEs, ALs for ACIs, and their corresponding CPs are reported in the second rows in all sample sizes.

## 7. Application to Real-Life Data

In this section, for illustrative purposes, real-life data are presented to inspect the inference procedures. We used two sets of data introduced by Badar and Priest [37] and used by Kundu and Gupta [2]. Set 1, denoted by (*X*) given in Table 9, is strength measured in GPA for single carbon fibers tested under tension at gauge lengths of 20 mm. Set 2, denoted by (*Y*) given in Table 10, is strength measured in GPA for single carbon fibers tested under tension at gauge lengths of 10 mm. Both Set 1 and Set 2 are of size 63. For the purpose of the goodness of fit test, the Kolmogorov–Smirnov (KS) distance between the empirical and the fitted distribution functions has been computed. It is 0.087588 and the associated *p* value is 0.7192 for Set 1, while it is 0.050055 and the associated *p* value is 0.9975 for Set 2. Hence, the *p* value for KS has the highest value for Sets 1 and 2. This leads us to conclude that WD is the best fit for the two real data sets. Empirical, *Q* − *Q*, and *P* − *P* plots are shown in Figures 3 and 4, which make it clear that the WD fits the data very well.

The article "Inferences for Stress-Strength Reliability Model in the Presence of Partially Accelerated Life Test to Its Strength Variable" was published in 2022. Journal: Comput Intell Neurosci.

Under the S-SPALT implementation on the strength variable *X*, the corresponding estimates of parameters change depending on the stress change time *τ*. For example, at *τ*=2.25 and *α*=2, MLEs of ${\hat{\beta }}_{1}=6.0934$, ${\hat{\beta }}_{2}=3.0594$, and $\hat{\lambda }=16.6242$. Thus, using (16), the MLE of *R* and its corresponding ACI is calculated as ${\hat{R}}_{\text{ML}}=0.48062$ and (0.38595, 0.57531) with length 0.18936, respectively. Also, by implementing the iterative algorithms mentioned in Section 4, the boot-p and boot-t CIs are computed as (0.33673, 0.52209) and (0.34746, 0.52972) with lengths 0.18536 and 0.18026.

Now, to compute the Bayesian estimate of *R*, the prior distributions of the parameters *β*_1_ and *β*_2_ are needed to specify. Because we have no prior information, we used the noninformative Gamma prior for *β*_1_ and *β*_2_ that is, the hyper-parameters are close to or equal to zero *a*_*i*_=0.0001 and *b*_*i*_=0.0001, *i*=1,2. Under the MCMC technique, the posterior analysis was done across combining MH algorithm within Gibbs sampler. To conduct the MCMC algorithm, which was described in Section 5, the initial values for the parameters *β*_1_, *β*_2_, and *λ* were taken to be their MLEs. In addition, 12000 MCMC samples were generated. To avoid the effect of the initial values, we expunge the first *β*_1_ samples as “burn-in.” Thus, the Bayesian estimate of *R* and its corresponding CRI is calculated as ${\hat{R}}_{\text{MC}}=0.47874$ and (0.34096, 0.51537) with length 0.17441, respectively.  Figure 5 displays 12000 chain values for *R*. The histogram and the kernel density estimate of *R* are shown in Figure 6. Also, we obtained more results with different values of *τ* as shown in Table 11.

## 8. Conclusions

In this paper, we consider the estimation of the stress-strength reliability model when the strength variable is subjected to the S-SPALT. By exposing the strength variable to the acceleration factor, a normal stress-strength model is forced to early failure; this design of the reliability has an effect on the level of reliability. We can illustrate it as follows: (i) In a specific stress change time, the increasing on acceleration loadings decreases the stress-strength reliability. (ii) Delaying stress change time helps maintain a level of reliability.

The article "Inferences for Stress-Strength Reliability Model in the Presence of Partially Accelerated Life Test to Its Strength Variable" was published in 2022. Journal: Comput Intell Neurosci.

The main aim of this paper is to study the effect of external stress loading on the strength variable. This external stress includes, for instance, temperature, voltage stress, thermal and electrical cycling and shock, vibration, mechanical stress, and radiation. Thus, the estimations of the stress-strength reliability model with the corresponding ACIs using the maximum likelihood, two parametric bootstrap, and Bayesian estimation methods are obtained. For illustrative purposes, we have applied a real-life example. A simulation study is computerized to inspect and compare the rendition of the proposed methods for different sample sizes (*n*, *m*), different acceleration factor *λ*, and different stress change time *τ*. From the results, we observe the following:

1. It is clear that, from Tables 1–8, as sample sizes (*n*, *m*) increase, the MSEs and average interval lengths decrease.
2. MLE, bootstrap, and Bayesian methods have very close estimates, and their ACIs have quite high CPs (around 0.95).
3. The ALs are decreasing with parallel to increasing on the actual value of *R*.
4. Bayes estimates perform better than the MLEs in terms of MSEs.
5. The ACIs of the MLEs have the smallest ALs, and the ACIs of the bootstrap-t have the largest ALs. At the same time, the Bayesian HPD intervals have the highest CPs.
6. Finally, we can conclude that the proposed inference methods give consistent results.
7. Sometimes, it is worth noting that the available data may be affected by uncertainties and/or inaccuracies. Then, strictly speaking, it would be necessary to carry out a fuzzy preprocessing of the data; see [38] as a future work.

## Figures and Tables

**Figure 1:** *R* values and corresponding *λ* values with increasing *τ* in the case of (*α*, *β*_1_, *β*_2_)=(2,0.4, 2).

**Figure 2:** *R* values and corresponding *τ* values with increasing *λ* in the case of (*α*, *β*_1_, *β*_2_)=(2,0.4, 2).

**Figure 3:** Empirical, Q-Q, and P-P plots of WD for Set 1.

**Figure 4:** Empirical, Q-Q, and P-P plots of WD for Set 2.

**Figure 5:** MCMC output of *R*.

**Figure 6:** Histogram of *R*.

**Table 1:** Means estimates of *R* (first row) with their MSEs (second row) and ALs (first row) for asymptotic, bootstrap, and HPD of *R* with their CPs (second row) in Case 1.

(*n*, *m*)	Point estimation		Interval estimation			
	${\hat{R}}_{\text{ML}}$	${\hat{R}}_{\text{MC}}$	ACI	boot − *p*	boot − *t*	CRI
(10,15)	0.75324	0.74654	0.67047	0.67288	0.69195	0.65232
	0.00667	0.00653	(0.9054)	(0.9123)	(0.9241)	(0.9436)
(20,25)	0.75841	0.74995	0.59351	0.58632	0.61472	0.60534
	0.00573	0.00564	(0.9147)	(0.9145)	(0.9345)	(0.9498)
(40,45)	0.76245	0.75942	0.45368	0.44564	0.47235	0.45214
	0.00457	0.00446	(0.9238)	(0.9324)	(0.9217)	(0.9524)
(60,60)	0.76349	0.76012	0.33452	0.32687	0.35647	0.34251
	0.00338	0.00325	(0.9417)	(0.9214)	(0.9356)	(0.9532)
(90,90)	0.76468	0.76219	0.21354	0.21000	0.23546	0.21344
	0.00213	0.00212	(0.9426)	(0.9335)	(0.9482)	(0.9547)

The article "Inferences for Stress-Strength Reliability Model in the Presence of Partially Accelerated Life Test to Its Strength Variable" was published in 2022. Journal: Comput Intell Neurosci.

**Table 2:** Means estimates of *R* (first row) with their MSEs (second row) and ALs (first row) for asymptotic, bootstrap, and HPD of *R* with their CPs (second row) in Case 2.

(*n*, *m*)	Point estimation		Interval estimation			
	${\hat{R}}_{\text{ML}}$	${\hat{R}}_{\text{MC}}$	ACI	boot − *p*	boot − *t*	CRI
(10,15)	0.82021	0.81988	**0.57013**	0.57227	0.63138	0.59241
	0.00622	0.00613	(0.9024)	(0.9185)	(0.9324)	(0.9428)
(20,25)	0.82152	0.82932	0.42635	0.43571	0.46354	0.44352
	0.00531	0.00520	(0.9354)	(0.9248)	(0.9245)	(0.9398)
(40,45)	0.82574	0.81873	0.35962	0.35441	0.37149	0.35912
	0.00407	0.00395	(0.9312)	(0.9187)	(0.9298)	(0.9425)
(60,60)	0.82648	0.81995	0.28874	0.28547	0.31645	0.29381
	0.00295	0.00271	(0.9399)	(0.9355)	(0.9358)	(0.9512)
(90,90)	0.82881	0.82116	0.20398	0.19564	0.21540	0.21011
	0.00183	0.00180	(0.9432)	(0.9452)	(0.9487)	(0.9501)

**Table 3:** Means estimates of *R* (first row) with their MSEs (second row) and ALs (first row) for asymptotic, bootstrap, and HPD of *R* with their CPs (second row) in Case 3.

(*n*, *m*)	Point estimation		Interval estimation			
	${\hat{R}}_{\text{ML}}$	${\hat{R}}_{\text{MC}}$	ACI	boot − *p*	boot − *t*	CRI
(10,15)	0.83023	0.82988	0.35341	0.36236	0.37138	0.35012
	0.00542	0.00539	(0.9188)	(0.9412)	(0.9314)	(0.9424)
(20,25)	0.83362	0.83179	0.29351	0.28952	0.31654	0.29551
	0.00410	0.00409	(0.9258)	(0.9289)	(0.9258)	(0.9432)
(40,45)	0.83012	0.83472	0.22348	0.21743	0.23452	0.23247
	0.00345	0.00347	(0.9314)	(0.9412)	(0.9347)	(0.9511)
(60,60)	0.82973	0.83147	0.16936	0.17638	0.18476	0.17325
	0.00255	0.00254	(0.9287)	(0.9384)	(0.9388)	(0.9521)
(90,90)	0.83362	0.82984	0.11084	0.10917	0.12331	0.11245
	0.00128	0.00129	(0.9425)	(0.9399)	(0.9481)	(0.9499)

**Table 4:** Means estimates of *R* (first row) with their MSEs (second row) and ALs (first row) for asymptotic, bootstrap, and HPD of *R* with their CPs (second row) in Case 4.

(*n*, *m*)	Point estimation		Interval estimation			
	${\hat{R}}_{\text{ML}}$	${\hat{R}}_{\text{MC}}$	ACI	boot − *p*	boot − *t*	HPD
(10,15)	0.82961	0.82247	0.34323	0.35001	0.36221	0.35221
	0.00523	**0.00522**	(0.9001)	(0.9264)	(0.9354)	(0.9532)
(20,25)	0.83213	0.82382	**0.27234**	0.26489	0.29652	0.28145
	0.00398	0.00399	(0.9254)	(0.9324)	(0.9136)	(0.9421)
(40,45)	0.82345	0.83347	0.20124	0.19999	0.22473	0.21003
	0.00332	0.00332	(0.9488)	(0.9455)	(0.9094)	(0.9542)
(60,60)	0.84998	0.83667	0.16210	0.16196	0.17235	0.17049
	0.00212	0.00211	(0.9378)	(0.9387)	(0.9324)	(0.9498)
(90,90)	0.83325	0.83471	0.10564	0.10588	0.11354	0.11134
	0.00111	0.00110	(0.9412)	(0.9541)	(0.9366)	(0.9493)

The article "Inferences for Stress-Strength Reliability Model in the Presence of Partially Accelerated Life Test to Its Strength Variable" was published in 2022. Journal: Comput Intell Neurosci.

**Table 5:** Means estimates of *R* (first row) with their MSEs (second row) and ALs (first row) for asymptotic, bootstrap, and HPD of *R* with their CPs (second row) in Case 5.

(*n*, *m*)	Point estimation			Interval estimation		
	${\hat{R}}_{\text{ML}}$	${\hat{R}}_{\text{MC}}$	ACI	boot − *p*	boot − *t*	CRI
(10,15)	0.30453	0.29547	0.24310	0.25834	0.26363	0.25549
	0.00282	0.00279	(0.9165)	(0.9134)	(0.9344)	(0.9475)
(20,25)	0.30145	0.30851	0.20154	0.21399	0.22632	0.21351
	0.00235	0.00228	(0.9226)	(0.9245)	(0.9481)	(0.9722)
(40,45)	0.31369	0.30658	0.15984	0.16541	0.18364	0.16543
	0.00186	0.00181	(0.9425)	(0.9219)	(0.9358)	(0.9655)
(60,60)	0.30487	0.29998	0.11369	0.12365	0.13841	0.11863
	0.00124	0.00117	(0.9344)	(0.9415)	(0.9410)	(0.9534)
(90,90)	0.29548	0.29963	0.08846	0.09476	0.10211	0.10254
	0.00089	0.00081	(0.9518)	(0.9424)	(0.9399)	(0.9714)

**Table 6:** Means estimates of *R* (first row) with their MSEs (second row) and ALs (first row) for asymptotic, bootstrap, and HPD of *R* with their CPs (second row) in Case 6.

(*n*, *m*)	Point estimation		Interval estimation			
	${\hat{R}}_{\text{ML}}$	${\hat{R}}_{\text{MC}}$	ACI	boot − *p*	boot − *t*	CRI
(10,15)	0.38369	0.37247	0.43215	0.44124	0.46278	0.43891
	0.00429	0.00425	(0.9021)	(0.9147)	(0.9247)	(0.9457)
(20,25)	0.37360	0.36981	0.35621	0.36452	0.38124	0.36112
	0.00361	0.00362	(0.9245)	(0.9025)	(0.9148)	(0.9542)
(40,45)	0.36961	0.37998	0.28352	0.29417	0.31254	0.29341
	0.00293	0.00289	(0.9199)	(0.9235)	(0.9365)	(0.9366)
(60,60)	0.37351	0.36457	0.21356	0.22458	0.23457	0.22154
	0.00214	0.00213	(0.9325)	(0.9471)	(0.9472)	(0.9547)
(90,90)	0.36543	0.36664	0.11347	0.13329	0.14328	0.12548
	0.00156	0.00155	(0.9398)	(0.9432)	(0.9398)	(0.9732)

**Table 7:** Means estimates of *R* (first row) with their MSEs (second row) and ALs (first row) for asymptotic, bootstrap, and HPD of *R* with their CPs (second row) in Case 7.

(*n*, *m*)	Point estimation			Interval estimation		
	${\hat{R}}_{\text{ML}}$	${\hat{R}}_{\text{MC}}$	ACI	boot − *p*	boot − *t*	CRI
(10,15)	0.31256	0.30647	0.29541	0.30584	0.31712	0.30097
	0.00372	0.00351	(0.9025)	(0.9035)	(0.9348)	(0.9641)
(20,25)	0.31131	0.31139	0.23752	0.24215	0.25136	0.24012
	0.00318	0.00315	(0.9184)	(0.9348)	(0.9412)	(0.9547)
(40,45)	0.31127	0.30694	0.18369	0.18985	0.19874	0.91414
	0.00249	0.00246	(0.9378)	(0.9254)	(0.9356)	(0.9523)
(60,60)	0.29987	0.29987	0.13258	0.13947	0.14692	0.13545
	0.00176	0.00168	(0.9501)	(0.9399)	(0.9188)	(0.9641)
(90,90)	0.30111	0.30654	0.09984	0.10564	0.12355	0.11021
	0.00099	0.00092	(0.9412)	(0.9410)	(0.9376)	(0.9752)

The article "Inferences for Stress-Strength Reliability Model in the Presence of Partially Accelerated Life Test to Its Strength Variable" was published in 2022. Journal: Comput Intell Neurosci.

**Table 8:** Means estimates of *R* (first row) with their MSEs (second row) and ALs (first row) for asymptotic, bootstrap, and HPD of *R* with their CPs (second row) in Case 8.

(*n*, *m*)	Point estimation		Interval estimation			
	${\hat{R}}_{\text{ML}}$	${\hat{R}}_{\text{MC}}$	ACI	boot − *p*	boot − *t*	CRI
(10,15)	0.36415	0.36931	0.48542	0.49548	0.50321	0.47632
	0.00454	0.00453	(0.9132)	(0.9199)	(0.9244)	(0.9573)
(20,25)	0.35989	0.36791	0.41562	0.43251	0.45567	0.42635
	0.00388	0.00389	(0.9245)	(0.9365)	(0.9523)	(0.9497)
(40,45)	0.36840	0.37113	0.33541	0.34564	0.36542	0.33988
	0.00317	0.00317	(0.9412)	(0.9274)	(0.9345)	(0.9584)
(60,60)	0.37465	0.36447	0.25356	0.27613	0.28941	0.26357
	0.00251	0.00249	(0.9348)	(0.9522)	(0.9388)	(0.9548)
(90,90)	0.36475	0.37894	0.13245	0.15328	0.16345	0.14571
	0.00176	0.00177	(0.9511)	(0.9463)	(0.9571)	(0.9612)

**Table 9:** Set 1 (*X*).

1.312	1.314	1.479	1.552	1.700	1.803	1.861	1.865	1.944	1.958	1.966	1.997
2.006	2.021	2.027	2.055	2.063	2.098	2.140	2.179	2.224	2.240	2.253	2.270
2.272	2.274	2.301	2.301	2.359	2.382	2.382	2.426	2.434	2.435	2.478	2.490
2.511	2.514	2.535	2.554	2.566	2.570	2.586	2.629	2.633	2.642	2.648	2.684
2.697	2.726	2.770	2.773	2.800	2.809	2.818	2.821	2.848	2.880	2.954	3.012
3.067	3.084	3.090									

**Table 10:** Set 2 (*Y*).

1.901	2.132	2.203	2.228	2.257	2.350	2.361	2.396	2.397	2.445	2.454	2.474
2.518	2.522	2.525	2.532	2.575	2.614	2.616	2.618	2.624	2.659	2.675	2.738
2.740	2.856	2.917	2.928	2.937	2.937	2.977	2.996	3.030	3.125	3.139	3.145
3.220	3.223	3.235	3.243	3.264	3.272	3.294	3.332	3.346	3.377	3.408	3.435
3.493	3.501	3.537	3.554	3.562	3.628	3.852	3.871	3.886	3.971	4.024	4.027
4.225	4.395	5.020									

**Table 11:** ML and Bayesian estimations with their lengths of the corresponding CIs for *R*.

	Point estimation			Approximate confidence lengths	
*τ*	${\hat{R}}_{\text{ML}}$	${\hat{R}}_{\text{MC}}$	ACI	boot − *p*	boot − *t*	CRI
1.5	0.51374	0.50179	0.29912	0.28301	0.27352	0.24364
2	0.50228	0.49367	0.30745	0.29810	0.28652	0.25632
2.5	0.44914	0.44134	0.17734	0.17054	0.16567	0.15234
3	0.40263	0.40019	0.15938	0.15069	0.14564	0.14842

## Data Availability

The article contains data generated from the statistical models used in the article.
